# Using Advanced Analytic Techniques to Optimize Cyber-Physical Defensive Plans in Sports Infrastructures and Facilities

**DOI:** 10.1155/2022/2061769

**Published:** 2022-06-11

**Authors:** Rui Wang

**Affiliations:** Zhengzhou Preschool Education College, Zhengzhou, Henan 450000, China

## Abstract

The technical projects for securing a network of infrastructures and processes are designed, financed, carried out, maintained, and operated within a general infrastructure system, which can gather activities and funds of the private or public sector. The importance of such projects for modern society is enormous, and there is a positive correlation between the size of infrastructure projects and the strength of the national economy. At the same time, it falls within the critical infrastructure sector most of the time. This work, taking into account the massive importance of investments made in the field of sports and the corresponding significance of the design and implementation of robust cybersecurity systems, presents an innovative optimization system for the design, performance, and adaptation of safeguards of technical projects, which require a high level of security standards. A realistic optimization system of low computational complexity is proposed and tested, dividing the problem into a series of subproblems of one-step optimization, which can be solved with great ease and without requirements on computational resources. The great innovation of the proposed system is that the separation is done so that the solution results from the optimal individual solutions of the subproblems without affecting the final result.

## 1. Introduction

The primary objective of programs to construct sports infrastructure is to be of service to, further advance, and generally better society. These activities include conceiving of, designing, constructing, and operating facilities necessary for contemporary sports culture and organizing and staging the relevant sporting events. These projects are an essential component of a nation's infrastructure and have significant repercussions on social and economic fronts [1]. They require significant capital investment, provide public services, and, in most cases, are considered to fall within the area of responsibility of the public sector. The necessity and feasibility of most of these projects are usually assessed by general methods of determining their economic characteristics (costs and benefits) [2, 3].

Professionals involved in sports infrastructure projects recognize the interdisciplinary nature of their design. In addition to the operational effectiveness of these projects and their impact on public cohesion, health, and security, planners are called upon to consider their beneficial and adverse environmental, social, and economic effects. They must also consider other factors (e.g., institutional, aesthetic, legal, and financial) to determine whether a particular project is safe and successfully implemented. Designers today are staffed with employees specialized in scientific fields, such as engineering, computer science, economics, and law, who, in addition to technical specialization, have a basic understanding of other sciences and the ability to work with other professionals because the implementation of these projects requires a high degree of interdisciplinarity, especially in the field of ensuring the infrastructure grid they cover [4].

In conclusion, the natural, environmental, social, and most importantly the security framework within which the design takes place varies from that of a patchwork of space-time and topographic elements. Therefore, while trying to adopt a broad strategy and comprehensive techniques, planners need to note that any unique athletic project provides a range of features and constraints. This is something that must be taken into consideration. Techniques that have been effectively implemented in the design process in the past for specific sports projects of varying sorts might serve as a reference for developing similar projects in the future. On the other hand, individuals in charge of the majority of the projects will probably be required to make modifications in response to the changing circumstances and the general security considerations that have to be taken into account.

This work presents an innovative optimization system for designing, performing, and adapting safeguards for technical projects requiring high-security standards. Taking into account the enormous importance of investments made in the field of sports and the corresponding significance of the design and implementation of robust cybersecurity systems, this work presents an innovative optimization system for the design, performance, and adaptation of safeguards. In particular, a cutting-edge and extremely realistic optimization system is proposed to be used to develop, implement, and maintain technical projects that call for a high level of security standards. The problem is broken down into a series of individual one-step optimization subproblems when using an analytical optimization system. These subproblems are much simpler and easier to solve than the original problem.

### 1.1. Related Literature Review

This section introduces the essential academic searches related to a practical approach to defending a cyber-physical system on technical and policy levels.

Mehrdad et al. [5] reviewed the publications on industrial cyber-physical security. They aimed to tackle the power transmission systems' protection strengths and vulnerabilities in the face of malicious assaults. They stated that to obtain a greater sense of protection for energy systems. When tackling energy network security issues, researchers should take a systematic approach and examine all phases of the holistic resilience cycle. To enhance the cyber-physical integrity of electrical power networks [6, 7], the idea of the Holistic Resilience Cycle was presented. This is a structured method to power system security that is defined by four steps (prevention and planning, detection, mitigation and reaction, and system recovery) as being inextricably linked and comprehensible only in context.

The study of Cai et al. [8] is characterized by attack modeling, security assessment, attack identification, and mitigation. Existing approaches were evaluated to ascertain the true nature of the cyber-physical power system security issue. Based on these technologies' features and evolution tendencies, the limits of the present research were identified, and solutions were proposed to further this field's study [9]. According to their security study, the future focal areas can be stated as follows: the field of theory to the offensive penetration method of systems should be examined in conjunction with the actual communication infrastructure and security prevention mechanisms. With the cyber and physical worlds inextricably linked, the power system cascade failure induced by cyberattacks was investigated, and a fusion analysis and quantitative risk assessment approach has been provided. Finally, attack modeling and defensive detection were accomplished using a cyber-physical fusion model. Then, following attack route prediction, a qualitative distinction of common defects and intense assaults, real-time assessment of protection stability, and digital aid decision-making could be accomplished.

Lai et al. [6] introduced a trilevel optimization model for constructing a coordinated assault scenario and determining the ideal defense strategy, which is novel in resource management to resist an attack. Additionally, considerable reductions in unsaved energy were seen when the suggested optimization technique was used to distribute defense resources. The numerical findings indicate that assault and defense methods vary according to offensive budgets, defense budgets, and restoration periods. Intruders are likely to conduct assaults that result in compounding failures, and the ideal defense approach would prevent such failures. Additionally, the formulation might be enhanced by factoring in the uncertainty associated with the attacker and restoration processes, dynamic difficulties, and grid storage incorporation.

He and Yan [2] conducted a thorough and systematic evaluation of significant smart grid attack risks and security measures. They began their assessment by providing an overview of smart grid security from a cyber-physical viewpoint before focusing on attack strategies that substantially influence the functioning of the power grid and the accompanying response measures. They then examined the potential problems associated with smart grid security after an in-depth examination of the threats and responses. They concentrated on assaults and defenses in the smart grid by conducting a complete and systematic analysis of the state-of-the-art in the sector, including everything from protection frameworks to attack methods and defensive techniques and a variety of possibilities and problems. They believed that their publication would inform people of attack dangers and mitigation techniques in complex cyber-infrastructure facilities such as the smart grid and would motivate researchers to work on developing secure and resilient networks.

Hao et al. [10] developed a strategy for effectively computing an execution plan that optimizes the number of engineered code iterations to achieve maximum protection impact while ensuring the guarded task system's real-time controllability through a novel reaction time analysis. They demonstrated how to incorporate protection mechanisms into practical cases. The suggested approach can determine a suboptimal plan for executing a designed operating security inspection code for shielded tasks or programs to obtain the maximum protection impact while ensuring the system's stimulability. Both simulation-based testing and an application of the suggested approach on a prototype self-driving vehicle demonstrate that the proposed method may be utilized to secure real-time systems.

Hasan et al. [11] provided a technique for prioritizing cyber risk remediation plans in cyber systems that are both efficient and cost-effective (safety implications). These researchers developed a framework for estimating how cyberattacks and random system failures could affect their security and cause catastrophic harm. We undertook an operational impact assessment to determine the magnitude of the damage caused by CPS threats. They advised constructing a model based on a data-driven attack and fault graph. In the end, they suggested building a strategic response decision capacity that comprises mitigation measures and policies that balance functional robustness and risk. The exploratory study in a real-world testbed showed that allocating resources based on node importance significantly decreased system-level risk. In the future, they were intending to expand the system and include all accessible system-level remediation measures, patch management, and system resilience.

### 1.2. Modeling the Cyber-Physical Defensive Plan

In modern reality, the complexity of systems and the evolution of technology require integrated defense security planning through an optimal economic approach [12, 13]. Existing experience shows that the anticipated benefits of such design are significant, especially in developing countries, in terms of the quality of the final result, the economy achieved, and the speed of implementation. This is the case even though the degree to which such methodologies are used varies depending on the type of project being undertaken. However, the rigorous application of the systemic concept in manufacturing technical works is a challenging endeavor. This is because it necessitates the detailed characteristics of the system, several technical-economic studies, the application of behavior calculation models, sensitivity analysis, and the formulation of optimal strategies regarding the objectives that have been established. Even though rigorous systematic studies could be beneficial, the abovementioned requirements render their implementation in small-scale projects impractical and prohibitive. However, decision-making is a necessary and ongoing process [6]. The development of systematic analysis techniques with simplified requirements, which most scholars accept and able to improve the effectiveness of promoted measures, is of great practical importance.

It should be noted that the mathematical models of the system in the method of systematic analysis play a central role in the modeling of the systems in question, as it is an essential tool in the modern design and management of projects and strategies [14, 15]. In general, such a model consists of one or more statements, expressed in mathematical terms, that describe relationships between dependent and independent variables, as shown in Figure 1.

The cyber-physical defensive plan is described with a mathematical model. This model is comprised of equations, logical assertions, and other instructions for processing the data that is currently available, as well as for creating and analyzing data that has been artificially generated [16]. The relationships that describe the system, correlating the input and output variables, are expressed by parameters, which are typically required to be determined by observations and measurements of the output variables and which can be constant or variable in a predetermined manner. In general, the parameters must be determined by the observations and measurements of the variables that are output from the system. Exogenous variables are those that the person experimenting does not have any influence over, and probability functions are used to characterize them. On the other hand, variables whose values can be entirely or partially determined are referred to as choice variables. These are the variables that are discussed further below. Restrictions or prohibitions that are applied to the model can include physical, economic, or any number of other factors that mathematical models can express [17, 18].

The analysis of mathematical models includes tables, graphs, mathematical equations, logical statements, and verbal descriptions, which are means of describing system boundaries, system input, and output elements and their relationships, and any feedback between output and input variables to achieve the desired result of the relevant modeling [19]. Specifically, the different types of mathematical models of the system depending on the types of mathematical functions used in this modeling are presented below [20, 21]:

(1) Algebraic equation: It can be obtained by adjusting a curve in empirical measurements; for example,
  (1) $$\begin{array}{c} y=f\left(x\right)=a_{0}+a_{1}x+a_{2}x^{2}. \end{array}$$
(2) Equation of differences: They can describe time-varying systems with delay, memory, multiple variables, and so on; for example,
  (2) $$\begin{array}{c} \frac{y_{k+1}=a_{k}y_{k}+b_{k}x_{k}}{z_{k+1}=\gamma_{1}y_{k+1}^{\gamma_{2}}}. \end{array}$$
(3) Normal differential equation: It can be obtained from processes of reduction or increase of the examined variable state; for example,
  (3) $$\begin{array}{c} \frac{\text{d}y}{\text{d}t}=ay\left(t\right)+bx\left(t\right), \end{array}$$
where *a*, *b* are the system parameters.
(4) Integral equation (an equation in which an unknown function appears under an integral sign): Known relationships that can be captured in the form of integral; for example,
  (4) $$\begin{array}{c} y\left(t\right)=\int_{t_{0}}^{t}g\left(t,\tau \right)x\left(\tau \right)\text{d}\tau . \end{array}$$
(5) Differential equation with some derivatives; for example,
  (5) $$\begin{array}{c} S\frac{\partial h}{\partial t}+\nabla \left(T\nabla h\right)=R-P, \end{array}$$
where *S*, *t*, *h*, *R*, *P* are the system parameters.

This particular equation is a differential equation, which means that it establishes a connection between one or more unknown functions and the derivatives of those functions. The function stands in for the system quantities; the results stand in for the rates of change those quantities are subject to, and the differential equation defines the connection between the two. To put it another way, the status variables represent the bare minimum of variables needed to describe the conditions of the system at any given time or location. Each possible configuration of the decision variables gives rise to a distinct policy or group of decisions. It is possible to implement a method if doing so does not violate any restrictions, and the area of viable approaches is the set of all possible policies taken together.

The objective function is an all-encompassing way of expressing various concepts related to optimality or the most desirable outcome. In a broader sense, the objective function is a performance indicator that we can use to evaluate the implications or derivatives produced by the system. For instance, the goal function can be utilized to calculate the cost of various amounts of resources generated or used in the context of the sports projects that are the topic of this conversation.

Summarizing the above, the methodology proposed for modeling the cyber-physical defensive plan requires [2, 11]:

(1) Model of the system in the general form (as described in Figure 1):
  (6) $$\begin{array}{c} \underline{y}=fn\left(\underline{x},\underline{u},\underline{\xi }\right), \end{array}$$
with
  (7) $$\begin{array}{c} \underline{y}={\left[y_{1},y_{2},\ldots y_{n}\right]}^{T},\\ \underline{x}={\left[x_{1},x_{2},\ldots x_{n}\right]}^{T},\\ \underline{u}={\left[u_{1},u_{2},\ldots u_{n}\right]}^{T},\\ \underline{\xi }={\left[\xi_{1},\xi_{2},\ldots \xi_{n}\right]}^{T}. \end{array}$$
(2) Performance indicator (objective function) related to the outcome of a specific policy applied to the problem:
  (8) $$\begin{array}{c} \min J=J\left(\underline{y},\underline{u}\right). \end{array}$$
(3) Set of restrictions:
  (9) $$\begin{array}{c} \frac{F\left(y,\underline{\text{u}}\right)=0}{G\left(y,\underline{\text{u}}\right)\geq 0}. \end{array}$$

It should also be emphasized that the system in question is thought of as a model of distributed parameters. This means that it takes into account the behavioral deviations from point to point throughout the system. This contributes to the system's overall complexity and the very realistic modeling that is followed. In addition, the primary modeling techniques can be broken down into four categories: statistical methods, research simulation using sampling techniques, probabilistic models and techniques, and modeling techniques based on probabilities.

### 1.3. Analytic Technique to Optimize Cyber-Physical Defensive Plan

After the cyber-physical defensive plan parametric system has been modeled, the general optimization problem is formulated as follows: we want to determine the values of the decision variables *u* that minimize the objective function *J* with known *J*, *F*, *G* functions under a set of constraints [22].

Specifically,

(10) $$\begin{array}{c} \text{min}J=J\left(\underline{y},\underline{u}\right),\\ F\left(\underline{y},\underline{u}\right)=0,G\left(\underline{y},\underline{u}\right)\geq 0. \end{array}$$

Decision theory is divided into two broad categories, based on whether the decision-maker is a single body or multiple bodies. So far, similar problems have been encountered in the first category of methods, which can be divided into static or single-stage and serial or multistage, where time can be discrete or continuous. The static problem concerns minimizing the cost function, which is a function of the decision variables vector. In the serial problem, the vector of system state variables evolves in time or space according to a method of equations in which decision variables are also involved. The cost function is the sum of the transition costs at each stage and ultimately depends on the (known) initial situation and values of the decision variables at each stage [14, 23]. The solution to the above problem for optimal control is developed using classical optimization methods where the functions are continuous and derivable without restrictions.

The proposed method is an advanced method that separates the multistage optimization problem into a series of single-stage optimization problems [24]. Even multistage systems of increased complexity, such as the one under consideration, can be solved with particular ease. The great innovation of the proposed solution is that the separation is done in such a way that the optimal solution of the initial problem results from the optimal solutions of the individual issues so that the method of solving does not affect the final result.

To be more specific, the following policy holds [25–27]:

(11) $$\begin{array}{c} \pi =\left\{\mu_{0},\ldots ,\mu_{N-1}\right\}, \end{array}$$

which is a set of functions that determines the values of the decision variables ${\underline{u}}_{k}$ from the values of the state variables ${\underline{x}}_{k}$; that is,

(12) $$\begin{array}{c} {\underline{u}}_{k}=\mu_{k}\left({\underline{x}}_{k}\right). \end{array}$$

The problem is to minimize costs for all possible policies *π* so that

(13) $$\begin{array}{c} {\text{min}}_{\pi }J_{\pi }\left({\underline{X}}_{0}\right)=J^{*}\left({\underline{X}}_{0}\right). \end{array}$$

Let *S*_*k*_ be the set of all possible states at time *k* so that

(14) $$\begin{array}{c} \left(S_{k}\subset R^{n}\right). \end{array}$$

And let *C*_*k*_ be the set of all possible decisions at time *k* so that

(15) $$\begin{array}{c} \left(C_{k}\subset R^{m}\right). \end{array}$$

For every

(16) $$\begin{array}{c} {\underline{x}}_{k}\in S_{k}⟺{\underline{u}}_{k}=\mu_{k}\left({\underline{X}}_{k}\right)\in C_{k}. \end{array}$$

Then, $U_{k}\left({\underline{X}}_{k}\right)$ is the sum of all possible decisions at time *k*, if the state is ${\underline{x}}_{k}$ (i.e., takes into account the constraints of the problem):

(17) $$\begin{array}{c} \left.U_{k}\left({\underline{X}}_{k}\right)\subset C_{k}\right). \end{array}$$

So, there is an acceptable policy:

(18) $$\begin{array}{c} \pi =\left\{\mu_{0},\ldots ,\mu_{N-1}\right\}, \end{array}$$

which is a set of functions that have a value field of the set:

(19) $$\begin{array}{c} U_{k}\left({\underline{x}}_{k}\right)or\mu_{k}:S_{k}⟶C_{k}. \end{array}$$

such that

(20) $$\begin{array}{c} \mu_{k}\left({\underline{X}}_{k}\right)\in U_{k}\left({\underline{X}}_{k}\right)\forall {\underline{X}}_{k}\in S_{k}. \end{array}$$

So, the intermediate cost depends only on the current situation at time *k* and takes the form

(21) $$\begin{array}{c} J_{k}\left(x_{k}\right)=g_{k}\left(x_{k},u_{k}\right)+J_{k+1}\left(f_{k}\left(x_{k},u_{k}\right)\right). \end{array}$$

In this equation, the problem of the existence of higher derivatives of the proposed function exists, where the sum of all possible decisions at time *k* is a function of the actual decision. An acceptable policy is a self-adjoint operator *π*, and *U* is a bounded self-adjoint operator. The proposed approach gives a new direction without multiple operator integrals to improve earlier results. It is a method that uses only unitary operators. This fact is proved as follows:

(22) $$\begin{array}{c} J_{N}=g_{N}\left(x_{N}\right)=J_{N}\left(x_{N}\right),\\ J_{N-1}=g_{N}\left(x_{N}\right)+g_{N-1}\left(x_{N-1},u_{N-1}\right)=g_{N-1}\left(x_{N-1},u_{N-1}\right)+J_{N}\left(x_{N}\right)\\ =g_{N-1}\left(x_{N-1},\mu_{N-1}\left(x_{N-1}\right)\right)+J_{N}\left(f_{N}\left(x_{N-1},\mu_{N-1}\left(x_{N-1}\right)\right)=J_{N-1}\left(x_{N-1}\right)\right.,\\ J_{N-2}=g_{N}\left(x_{N}\right)+g_{N-1}\left(x_{N-1},u_{N-1}\right)+g_{N-2}\left(x_{N-2},u_{N-2}\right)=g_{N-2}\left(x_{N-2},u_{N-2}\right)+J_{N-1}\left(x_{N-1}\right)\\ =g_{N-2}\left(x_{N-2},\mu_{N-2}\left(x_{N-2}\right)\right)+J_{N-1}\left(f_{N-1}\left(x_{N-2},\mu_{N-2}\left(x_{N-2}\right)\right)\right)=J_{N-2}\left(x_{N-2}\right). \end{array}$$

And the problem of minimization at each stage is expressed as follows:

(23) $$\begin{array}{c} J_{N}^{*}\left(x_{N}\right)=g_{N}\left(x_{N}\right),\\ J_{k}^{*}\left(x_{k}\right)={\text{min}}_{u_{k}\in U_{k}\left(x_{k}\right)}\left[g_{k}\left(x_{k},u_{k}\right)+J_{k+1}^{*}\left(f_{k}\left(x_{k},u_{k}\right)\right)\right],\\ k=N-1,N-2,\ldots ,0, \end{array}$$

where *J*_*k*_^*∗*^(*X*_*k*_)=*J*^*∗*^(*X*_*k*_) is the optimal cost for the problem starting from the state *x*_*k*_ at time *k* and thus *J*_0_^*∗*^(*X*_0_)=*J*^*∗*^(*x*_0_) is the minimum cost of transition from *x*_0_ to *x*_Ν_:

Consequently, if

(24) $$\begin{array}{c} \exists \pi^{*}=\left\{\mu_{0}^{*},\ldots ,\mu_{N-1}^{*}\right\}, \end{array}$$

such that

(25) $$\begin{array}{c} \mu_{k}^{*}\left(X_{k}\right), \end{array}$$

achieves the minimum for each *X*_*k*_; then, *μ*^*∗*^ is the optimal policy because

(26) $$\begin{array}{c} J_{N}^{*}\left(x_{N}\right)=g_{N}\left(x_{N}\right), \end{array}$$

which is calculated from

(27) $$\begin{array}{c} J_{k}\left(x_{k}\right)=g_{k}\left(x_{k},u_{k}\right)+J_{k+1}^{*}\left(x_{k+1}\right). \end{array}$$

So, based on the principle of optimality, if {*μ*_0_^*∗*^,…, *μ*_*N*−1_^*∗*^} is optimal for the initial problem, then {*μ*_*k*_^*∗*^,…, *μ*_*N*−1_^*∗*^} is optimal for the problem starting at time *k*.

Finding the most effective approach to solving many important practical problems requires one to investigate many approaches. In many cases, this requires determining either the highest or lowest value that can be returned by a function. The majority of these issues can be resolved by first locating the right function and then applying the principles of calculus in order to ascertain whether the needed maximum or minimum value should be found. In this problem, this means that the best policy will yield the minimum cost of moving to the final state from any intermediate stage *k*. The proof of this is based on the following two propositions [28]:

(28) $$\begin{array}{c} {\text{min}}_{x,y}\left[h_{1}\left(x\right)+h_{2}\left(x,y\right)\right]={\text{min}}_{x}\left[h_{1}\left(x\right)+{\text{min}}_{y}h_{2}\left(x,y\right)\right]. \end{array}$$

(29) $$\begin{array}{c} {\text{min}}_{\mu }\left[h\left(x,\mu \left(x\right)\right]={\text{min}}_{\mu }\left[h\left(x,u\right)\right].\right.. \end{array}$$

As for *i* + 1,

(30) $$\begin{array}{c} j_{i+1}^{*}\left(x_{i+1}\right)=j^{*}\left(x_{i+1}\right)=\min_{\left\{\mu_{i+1},\ldots ,\mu_{N-1}\right\}}\left[g_{N}\left(x_{N}\right)+\sum_{k=i+1}^{N-1}g_{k}\left(x_{k},\mu_{k}\left(x_{k}\right)\right)\right]. \end{array}$$

Then, for *i*, we have

(31) $$\begin{array}{c} J^{*}\left(x_{i}\right)={\text{min}}_{\left\{\mu_{i},\ldots ,\mu_{N-1}\right\}}\left[g_{N}\left(x_{N}\right)+\sum_{k=i}^{N-1}g_{k}\left(x_{k},\mu_{k}\left(x_{k}\right)\right)\right]. \end{array}$$

So,

(32) $$\begin{array}{c} =\min_{\mu_{i}}g_{i}\left(x_{i},\mu_{i}\left(x_{i}\right)\right)+\min_{\left\{\mu_{+1},\ldots ,\mu_{k+1}\right\}}\left[g_{N}\left(x_{N}\right)+\sum_{k=i+1}^{N-1}g_{k}\left(x_{k},\mu_{k}\left(x_{k}\right)\right)\right]\\ =\min_{\mu_{i}}g_{i}\left(x_{i},\mu_{i}\left(x_{i}\right)\right)+J^{*}\left(x_{i+1}\right)\\ =\min_{\mu_{i}}g_{i}\left(x_{i},\mu_{i}\left(x_{i}\right)\right)+J^{*}\left(x_{i+1}\right). \end{array}$$

And so,

(33) $$\begin{array}{c} ={\text{min}}_{u_{i}\in U_{i}\left(x_{i}\right)}g_{i}\left(x_{i},u_{i}\right)+J_{i+1}^{*}\left(f_{i}\left(x_{i},u_{i}\right)\right)=J_{i}^{*}\left(x_{i}\right). \end{array}$$

This fact verifies the request and solves the initial optimization problem.

Finally, although the computational load can be huge for a large number of decision variables and many stages, the proposed algorithm |*C*| × |*S*| × *N* is much faster than the simple solutions. As shown above, no exhaustive calculation is applied for each *k*, provided that

(34) $$\begin{array}{c} S_{k}⟶C_{k}|Cl^{\left|S\right|}. \end{array}$$

Since for *N* stages, the policy *π*={*μ*_0_,…, *μ*_*N*−1_} is optimized based on

(35) $$\begin{array}{c} {\left\{{\left|C\right|}^{\left|S\right|}\right\}}^{N}={\left|Cl\right|}^{\left|S\right|N}. \end{array}$$

Lattice models are a method that can be utilized in the valuation of economic derivatives. In a lattice model, the shortest route is searched to make the best conclusion on finding the most inexpensive bid in the search for CCTV equipment for the physical perimeter security of the sports project under consideration. It is necessary to use a discrete-time model to model the potential correlation aspects of complicated issues. The preceding technique is shown using a concrete case described in detail [29–31]. Due to the dependence on multiple paths, the Monte Carlo methods fail to make optimal decisions. The Monte Carlo methods are a comprehensive class of computer algorithms based on the concept of repeatedly taking a sample from a random pool to acquire numerical results. The fundamental idea is to use a chance to find solutions to problems that, in theory, might be solved using deterministic methods. When the issue in question involves a large number of variables that are each constrained uniquely, these methods are computationally inefficient. This indicates that approximating a solution using these methods consumes a significant amount of both time and computational effort. In addition, the model will produce unsatisfactory outputs if the parameters and constraints that are fed into it are of low quality. In this example, the solution with the minimum cost is requested within the A–Z, where the transition costs are as shown in Figure 2.

As shown in the figure, no loop has a negative cost. If the connection *ij* does not exist we set *c*_ij_ = infinity, while *c*_*ii*_ is taken as 0. Also, *x*_k_ is taken as the state where the node is in *k* stage (stage is the transition between nodes, and control is the decision of the next situation). *X*_*k*+1_=*u*_*k*_ is taken as a dynamic equation, and *g*_*k*_(*X*_*k*_, *u*_*k*_)=*c*_*X*_*k*__*u*_*k*_=*c*_*ij*_ as a cost function.

So based on the proposed algorithm, we have

(36) $$\begin{array}{c} J_{N}\left(x_{N}\right)=g_{N}\left(x_{N}\right)=\left\{\frac{\infty \;if\;x_{N}=A}{0\;if\;x_{N}=Z}.\right. \end{array}$$

The optimal cost to get to node *j* starting from *i* is calculated as follows:

(37) $$\begin{array}{c} J_{k}\left(x_{k}\right)={\text{min}}_{u_{k}}\left[c_{x_{k}u_{k}}+J_{k+1}\left(u_{k}\right)\right]\eta J_{k}\left(i\right)={\text{min}}_{j}\left[c_{ij}+J_{k+1}\left(j\right)\right]. \end{array}$$

Implementing the corresponding table of statements, without using exhaustive calculation, the statements are calculated as follows [32–34]:

(38) $$\begin{array}{c} 3^{3}=n^{N-1}\text{where }N\geq 3, \end{array}$$

where *N* is the number of stages and *n* is the number of nodes in each intermediate stage.

The solution will occur in 3 stages, wherein each stage a decision will be made for an offer. The benefits are

(39) $$\begin{array}{c} a_{j}\left(1-e^{-b_{j}x_{j}}\right). \end{array}$$

The costs are

(40) $$\begin{array}{c} c_{j}x_{j}^{d_{j}}. \end{array}$$

The state equation is

(41) $$\begin{array}{c} S_{j+1}=S_{j}-X_{j}. \end{array}$$

The objective function is

(42) $$\begin{array}{c} g_{j}\left(x_{j}\right)=a_{j}\left(1-e^{-b_{j}x_{j}}\right)-c_{j}x_{j}^{d_{j}}. \end{array}$$

So,

(43) $$\begin{array}{c} \frac{J_{N}^{*}\left(S_{N}\right)=g_{N}\left(S_{N}\right)=0}{J_{j}^{*}\left(X_{j}\right)={\text{max}}_{x_{j}}\left[g_{j}\left(x_{j}\right)+J_{j+1}^{*}\left(S_{j}-X_{j}\right)\right]j=N-1,N-2,\ldots ,0}. \end{array}$$

Therefore, the best policy is

(44) $$\begin{array}{c} \frac{A\left[10\right]⟶B_{1}\left[8\right]⟶C_{1}\left[8\right]⟶D_{1}\left[9\right]⟶Zf^{*}=35}{A\left[10\right]⟶B_{1}\left[9\right]⟶C_{3}\left[7\right]⟶D_{1}\left[9\right]⟶Zf^{*}=35}. \end{array}$$

## 2. Conclusions

In this work, we proposed an innovative optimization system for designing, implementing, and updating technical security projects, which require a high level of security standards. It is an analytical way of optimizing that divides the multistage optimization problem into a series of one-step optimization problems. Even multistage systems of increased complexity can be solved with particular ease. The great innovation of the proposed solution is that the separation is done in such a way that the optimal solution of the initial problem results from the optimal solutions of the individual issues so that the method of solving does not affect the result.

A clear example of the proposed procedure was presented descriptively. Specifically, the shortest route was sought in a lattice model to find the best decision on finding the most economical bid in the search for CCTV equipment for the physical perimeter security of the sports project in question. The solution with the minimum cost was achieved based on the proposed approach.

The extensive comparison with probabilistic methodologies that represent parts of stochastic systems through appropriate statistical parameters is an essential aspect that they should expand upon in the next stage of this research project. Additionally, queuing methods and inventory theory may give models for more extensive optimization and perhaps more efficient local decision-making systems.

## Figures and Tables

**Figure 1:** Schematic description of the mathematical model.

**Figure 2:** Financial lattice model.

## Data Availability

The data used in this study are available from the corresponding author upon request.
